RETRACTED

# Acupuncture Enhances Gastrointestinal Motility and Improves Autonomic Nervous Function in Patients with Septic Gastrointestinal Dysfunction

**DOI:** 10.1155/2022/1653290

**Published:** 2022-09-21

**Authors:** Lihong Ban, Yongpeng Pu, Huanyuan Huang, Bin You, Wei Chen, Yanzhen Wang

**Affiliations:** ^1^Department of Critical Medicine, The First People's Hospital of Lanzhou City, Lanzhou, Gansu 730050, China; ^2^Department of Clinical Laboratory, The First People's Hospital of Lanzhou City, Lanzhou, Gansu 730050, China; ^3^Department of Rehabilitation Medicine, The First People's Hospital of Lanzhou City, Lanzhou, Gansu 730050, China

## Abstract

Gastrointestinal dysfunction (GD) is a common complication after endotoxemia, which can further aggravate the progress of infection. Acupuncture uses metal needles of different shapes and techniques to stimulate specific points on the human body, which are effective in treating various diseases, including gastrointestinal diseases. We aimed at exploring the clinical effect of acupuncture on the recovery of visceral sensation, proximal gastric compliance, and autonomic nervous function in patients with septic GD. A total of 73 sepsis with GD patients were selected using modified single section ultrasonography combined with clinical symptoms in the First People's Hospital of Lanzhou City during 2019. The participants were randomly allocated to routine-treatment (control group) and study group receiving acupuncture. The indexes before and after treatment included gastric residue, gastric dilatation, pressure and volume, gastric compliance, autonomic nerve function, APACHE II score, and infection index were measured and compared. Before treatment, there was no significant difference in the basic information of the two groups, including gastric volume and pressure, gastric residue, gastric compliance, autonomic nerve function, and APACHE II score. After treatment, the maximum gastric volume and pressure, gastric residue, and APACHE II score of the two groups were significantly improved (*P* < 0.05). In addition, the maximum gastric volume and pressure of the study group were significantly higher, while gastric residual, autonomic nerve function, and APACHE II were significantly lower than those of the control group (*P* < 0.05). However, our results showed that acupuncture did not further reduce inflammatory markers, including white blood cells, C-reactive protein, and procalcitonin. To sum up, on the basis of basic treatment, the application of acupuncture can further improve the clinical symptoms of GD in patients with sepsis, enhance gastrointestinal motility, and improve autonomic nervous function, which is worthy of clinical application and promotion.

RETRACTED

## 1. Introduction

Sepsis causes homeostasis imbalance and leads to multiple organ dysfunction, which determines its high risk and refractory [1, 2]. Gastrointestinal tract is the main target organ and “stress response center” of sepsis. Gastrointestinal dysfunction (GD) is the most common and important prognostic factor in multiple organ dysfunction syndrome (MODS) [3]. Similarly, GD is also the “starting organ”, which can expand the inflammatory response and affect the prognosis of sepsis [4]. GD induced by sepsis is a clinical manifestation that involves impaired gastrointestinal function after the systemic inflammatory response caused by infection, and is one of the essential causes of exacerbation and death in critically ill patients [5]. In addition, gastrointestinal dysfunction in sepsis accounts for a large proportion of MODS, with a high morbidity and mortality rate, and an extremely poor prognosis [6]. Therefore, actively improving the gastrointestinal function of patients is of great significance to improve the success rate of sepsis treatment.

For GD, the current western medicine treatment mode is mainly based on its etiology and clinical symptoms, such as antidiarrheal, analgesic, laxative, and promoting gastric motility [5]. However, there are still some patients with GD eventually leading to further deterioration of infection [7]. In recent years, traditional Chinese medicine treatment has been proved to have significant improvement effect in the study of gastrointestinal function in patients with sepsis [6, 8]. Therefore, to explore the characteristic therapy of traditional Chinese medicine and to use the advantages of traditional Chinese medicine to treat this disease has broad prospects and important significance.

Currently, a large number of studies have found that acupuncture plays an important role in gastrointestinal motility [7, 9]. Acupuncture, as the most commonly used technique in traditional Chinese medicine, mainly uses metal needles of different shapes and different techniques to stimulate certain acupoints on the human body. Through the channels and acupoints, adjust the human body viscera qi to achieve the purpose of treatment [10]. It has been reported that acupuncture can promote the recovery of gastrointestinal function in patients with GD after abdominal surgery on the basis of conventional western medicine treatment [11]. Also, acupuncture can reduce the systemic inflammatory response of patients with sepsis, promote the recovery of body functions, and improve clinical symptoms and prognosis. Acupuncture has a significant improvement effect on GD induced by sepsis, which mainly focuses on 2 aspects: inhibition of inflammation and immune promotion.

RETRACTED

Based on previous studies, our aim is to confirm therapeutic effect of acupuncture in patients with septic GD. The indexes included gastric residue, gastric dilatation, pressure and volume, gastric compliance, autonomic nerve function, acute physiology, and chronic health evaluation II (APACHE II) score and infection index were detected before and after treatment. This study will provide further evidence as to whether acupuncture should be included in enhanced recovery for patients with septic GD.

## 2. Methods

### 2.1. Study Design

This study is a prospective, observational, and randomized control trial. It was conducted in 2019 and approved by the Ethics Committee of the First People's Hospital of Lanzhou City (approval number: G2019-7). All procedures were performed in accordance with the relevant guidelines and regulations. Informed consent forms have been obtained from all representatives of the patients.

### 2.2. Patients

A total of 73 patients with septic GD were selected from the First People's Hospital of Lanzhou City and randomly divided into control group (*n* = 36) and study group (*n* = 37) [12]. Inclusion criteria: (1) conform to the diagnosis criteria of sepsis as proposed in the Third International Consensus Definitions for Sepsis and Septic Shock (Sepsis-3) [13]]; (2) conform to the diagnostic criteria of GD grade II-III; (3) patients and their families received acupuncture treatment. Exclusion criteria: (1) did not meet the diagnostic criteria of sepsis and GD grade II-III; (2) mental disorders, pregnant women, or lactating women; (3) ICU stay < 3 days; (4) ≤18 years of age; (5) esophagus, stomach, or intestinal medical and surgical histories or primary injury to the gastrointestinal tract; (6) patients and their families were unwilling to receive acupuncture treatment. There were 18 males and 18 females in the control group, with an average age of 70.32 ± 8.58 years old. In the study group, there were 19 males and 18 females, with an average age of 70.22 ± 9.14 years old. There was no significant difference in gender or age between the two groups.

### 2.3. Determination of White Blood Cells (WBC), C-Reactive Protein (CRP), and Procalcitonin (PCT) Levels

After 8 h of fasting, 5 ml of fasting peripheral venous blood was collected from the patient, and the samples were immediately tested on the machine for CRP and PCT. The WBC count was performed using a Glitter GRT-6001 hematology analyzer. CRP level was evaluated using Myriad BC5390 fully automated hematology analyzer for latex-enhanced immunoturbidimetric assay. PCT assay was conducted using Radiometer AQT90 rapid immunoassay and time-resolved fluorescence immunoassay.

RETRACTED

### 2.4. Ultrasonic

The modified single section method of gastric antrum was used for obtaining the contraction area of gastric antrum of patients before and after treatment of acupuncture. The superior mesenteric vein, the abdominal aorta, and the left lobe of the liver were used as sinusoidal landmarks, and the sinusoids were probed at the mid-upper abdominal body surface landmark points to determine the size of the sinusoidal area during fasting. The gastric cavity was filled with warm water orally in healthy subjects and via gastric tube in critically ill patients. The maximum diastolic area of the gastric sinus was measured immediately after filling, and then repeated every 5 minutes until the liquid dark area in the stomach disappeared, which was the gastric emptying time (GET).

### 2.5. Treatments

On the basis of anti-infection and organ function support treatment, the control group was treated with gastrointestinal motility drugs. Referring to the International Guidelines for the Treatment of Sepsis and Infectious Shock (2016), the treatment for the control group included: (1) organ support treatment by ventilator, hemofiltration, and vasoactive drugs to maintain basic vital signs; (2) symptomatic treatment such as fluid resuscitation and anti-infection; (3) protection of the gastrointestinal barrier mucosa when GD occurred; (4) regulation of microecology, improvement of intestinal microcirculation, and reduction of gastrointestinal mucosal permeability; and (5) symptomatic support treatment such as strengthening enteral nutrition and promoting gastrointestinal motility.

In contrast, on the basis of anti-infection and organ function support treatment, the study group was given an acupuncture treatment. Acupuncture will be performed by a licensed acupuncturist who holds a China Acupuncturist Certification, with at least 2 years of clinical experience in acupuncture. Acupuncture points included Shangwan, Zhongwan, Xiawan, bilateral Tianshu, Guanyuan, Qihai, bilateral Zusanli, and bilateral Gongsun. Both groups were observed for 1 week. The needle used is ‘Hua Tuo brand' disposable sterile needles, with diameter 0.30 mm and length 40 mm, the manufacturer is Suzhou Medical Supplies Factory Co. The site of insertions will be swabbed and disinfected with 75% alcohol before needle insertion.

Shangwan is located in the Ren channel. It is the meeting point with the foot yangming stomach meridian and the hand sun small intestine meridian and has the function of strengthening the spleen and stomach, and of clearing and distributing turbidity. Positioned on the anterior median line, 5 inches above the umbilicus; the operation is to pierce 1 inch directly and retain the needle for 30 minutes.

RETRACTED

Zhongwan is located in the Ren channel, and is a point of the foot yangming stomach, and a point of the eight Hui points of the internal organs, with the effect of tonifying the middle and benefiting the qi, raising the clear, and lowering the turbid denial. Positioned on the front median line, 4 inches above the umbilicus, or at the midpoint of the joint line between the umbilicus and the thoracic sword; the operation is to pierce 1 inch directly and keep the needle for 30 minutes.

Xiawan is located in the Ren vessel, it is a meeting point with the foot taiyin spleen meridian and has the function of transporting and raising the clear. It is positioned on the front median. It is located on the anterior midline, 2 inches above the umbilicus; the operation is to pierce 1 inch directly and keep the needle for 30 minutes.

Bilateral tianshu isocated in the foot yangming stomach meridian, it is a point of the large intestine, with the effect of clearing turbidity from the internal organs. Positioned at 2 inches next to the middle of the umbilicus; the operation is to pierce 1 inch directly and retain the needle for 30 minutes.

Bilateral zusanli is a joint point of the foot yangming stomach meridian and is the lower joint point of the foot yangming stomach, which can be tonified if the spleen and stomach are deficient. It is positioned at the calvaria point (flexed knee, in the lateral recess of the patellar ligament. It is located 3 inches below the calvaria point (in the lateral recess of the patellar ligament), 1 finger outside the anterior tibial crest; the operation is to pierce 1 inch directly and retain the needle for 30 minutes.

Guan Yuan is on the midline of the abdomen, three inches below the umbilicus, and the midpoint from the Guanyuan to the navel is the Qihai; the operation is to pierce 1 inch directly and retain the needle for 30 minutes.

Bilateral Gongsun is located on the medial edge of the foot, just below the base of the first metatarsal; the operation is to pierce 1 inch directly and retain the needle for 30 minutes.

### 2.6. Adverse Events

If some adverse events including severe convulsions pain were caused by acupuncture intervention, aggravating symptoms, or other critical diseases occur during treatment and cannot be continued, the researchers found serious safety problems, as well as patients cannot stick to treatment for a variety of reasons, the patients will be dropped out of the study.

### 2.7. Observed Indexes

1. The indexes, including the initial and maximal pressure and volume, symptom scores under different gastric dilatation volumes and gastric compliance were obtained with the Synectice Visceral Stimulator (SVS)/Barostat before and 1 week after the treatment. Bamstat can maintain the set pressure or volume level through electronic feedback mechanism, and measure the corresponding changes of gas volume or pressure in the airbag. SVS/Barostat was used for isovolumic mechanical gastric distention; 50 ml volume was increased every 2 minutes from 0. The symptom scores of abdominal distension, epigastric pain, nausea, and vomiting were recorded when the volume was 200 ml, 300 ml, and 400 ml, respectively. Each symptom was divided into 0-3 points (0 = no symptom, 1 = mild symptom, need attention to feel the symptom exists, 2 = moderate symptom, can feel the symptom exists, but can tolerate, 3 = severe symptom, unbearable). At the same time, the initial volume (the volume at which the subject began to feel discomfort or fullness in the upper abdomen when receiving the stimulation of gastric distention) and the maximal volume (the volume at which the subject began to feel pain or unbearable in the upper abdomen when receiving the stimulation of gastric distention) were recorded, as well as the corresponding initial pressure and maximal pressure. Besides, automatically generated gastric compliance was also recorded
2. Autonomic nervous function was evaluated as followed. In brief, 15 minutes electrocardiograph (ECG) was recorded as baseline ECG. Then, isovolumic mechanical gastric dilatation was performed by barostat, and when the volume of gas injected into the balloon reached the maximum tolerated volume, 15 minutes ECG was recorded in the study group and the control group. After then, in the study group, acupuncture was performed for 20 minutes, and ECG was recorded 15 minutes after acupuncture. While in the control group, acupuncture was not performed, and the ECG was recorded for 15 minutes. Heart rate variability analysis indexes, including low frequency (LF: 0.04-0.15 Hz), high frequency (HF: 0.15-0.40 Hz), and very low frequency (VLF: below 0.03 Hz) were calculated at baseline in the maximal tolerance state and after acupuncture, respectively
3. APACHE II score was calculated with the worst physiologic parameters during the first 24 hours before and after treatment to measure the clinical severity of each patient's objective physical condition upon presentation [14]

RETRACTED

### 2.8. Statistical Methods

SPSS 22.0 was used for statistical analysis. The measurement data were expressed by (mean ± standard deviation) and compared with analysis of variance. *P* < 0.05 meant the difference was significant.

## 3. Results

### 3.1. Application of Ultrasonic Modified Single Section of Gastric Antrum in the Diagnosis of Patients with Septic GD

The modified single section method of gastric antrum can be used for the diagnosis of patients with septic GD by obtaining the contraction area of gastric antrum. As shown in Figure 1(a), before acupuncture, result of ultrasonography indicates the increased contraction area of the gastric antrum. After acupuncture for two days, the contraction area of the gastric antrum was decreased compared with that before acupuncture treatment (Figure 1(b)). After acupuncture for five days, the contraction area of the gastric antrum was further decreased and was basically restored to a normal condition (Figure 1(C)).

Before treatment (−1 and 0 days), both groups had significant delayed gastric emptying (defined as gastric residual volume (GRV)s ≥ 500 ml, lasting for ≥ 2 days). Compared with the results of GRVs on the day of treatment, GRVs of the two groups were significantly decreased after treatment (*P* < 0.001). In addition, compared with the control group, GRVs in the study group reduced more significantly after treatment (*P* < 0.01 and *P* < 0.001), as shown in Figure 2.

### 3.2. Comparison of the Initial and Maximal Pressure and Volume between the Two Groups

Before treatment, there was no significant difference in initial pressure and initial volume between the study group and the control group. After treatment, the initial pressure and initial volume of the two groups both increased, and the study group increased more (*P* < 0.05). Besides, before treatment, there was no significant difference in maximal pressure and maximal volume between the study group and the control group. After treatment, the maximal pressure and maximal volume of the two groups both increased, and the study group increased more (*P* < 0.05), as shown in Table 1.

### 3.3. Comparison of Symptom Scores under Different Gastric Dilatation Volumes between the Two Groups

Before treatment, when the expansion volume was 200 ml, 300 ml, and 400 ml, there was no significant difference in symptom scores (including epigastric pain, fullness, and nausea or vomiting) between the two groups. However, after treatment, when the expansion volume was 200 ml, 300 ml, and 400 ml, the symptom scores of the two groups all decreased, and the decrease of the study group was more obvious (*P* < 0.05), as shown in Table 2.

### 3.4. Comparison of Gastric Compliance between the Two Groups

Before treatment, there was no significant difference in gastric compliance between the study group and the control group (*P* > 0.05). After treatment, the gastric compliance of the two groups both improved, and the improvement of the study group was more obvious (*P* = 0.0033 and *P* < 0.0001), as shown in Table 3.

RETRACTED

### 3.5. Effect of Acupuncture on Autonomic Nervous Function in Patients with Septic GD

Compared with baseline state, the HF in the maximal tolerance state showed a downward trend (*P* < 0.05), which indicated that expansion could reduce the HF, that was, the tension of vagus nerve; while the LF and VLF in the maximal tolerance state showed an upward trend (*P* < 0.05), which indicated that expansion could increase the LF and VLF, that was, the tension of sympathetic nerve. However, acupuncture could adjust the downward trend of HF and the upward trend of LF and VLF caused by gastric distention, that was, acupuncture could adjust the downward trend of vagus nerve tension and the upward trend of sympathetic nerve tension caused by gastric distention, so as to improve vagus nerve tension and reduce sympathetic nerve tension, as shown in Table 4.

### 3.6. Comparison of APACHE II Score, Abdominal Circumference and Intraperitoneal Pressure between the Two Groups

After treatment, APACHE II score and intraperitoneal pressure were lower in both groups than before treatment, and the improvements of the study group were more obvious than those of the control group (*P* < 0.05). However, there was no significant difference in abdominal circumference between the two groups before and after treatment, as shown in Table 5.

Comparison of infection indexes between the two groups.

After treatment, WBC, CRP, and PCT in both groups were significantly decreased (*P* < 0.05), but acupuncture could not further reduce these inflammatory indexes, as shown in Table 6.

## 4. Discussion

GD is one of the main manifestations of multiple organ dysfunction syndrome (MODS) caused by sepsis [15, 16]. Its clinical manifestations are abdominal distension, vomiting, and diarrhea caused by more gastric residues, as well as intestinal dyskinesia, stress ulcer, and gastrointestinal bleeding [17]. When these symptoms appear at the same time, the mortality of patients can be significantly increased [3]. GD caused by sepsis is mainly mediated by inflammation, which can destroy the integrity of intestinal epithelium and the ability of immune response, leading to GD [18]. In addition, the inflammatory reaction can also increase the intestinal permeability, leading to bacteria passing through the intestinal wall, promoting the further development of sepsis, forming a vicious circle [19].

Weakness of spleen and stomach is the pathogenesis of GD in sepsis, often accompanied by fatigue, anorexia, pale complexion, palpitations, chest tightness, shortness of breath, excessive sweating, and other symptoms [20]. These phenomena of spleen and stomach weakness can be fundamentally improved by tonifying the spleen and stomach, supporting healthy qi, strengthening the main body, and fighting the enemy “syndrome differentiation and treatment, overall regulation” is an important principle of TCM treatment of diseases [21, 22]. In this study, we selected patients with GD in the late stage of sepsis, most of them were weak in spleen and stomach, sepsis patients were in a high metabolic state, and metabolic pathways were abnormal. If at this time the spleen and stomach function is damaged, the blood biochemical source is deficient, the patient's nutritional status is low, the healthy qi is deficient, and the human body's ability to remove pathogenic factors is reduced, thus prolonging the course of sepsis.

RETRACTED

The essence of acupuncture is to stimulate healthy qi by triggering and strengthening the body's homeostasis function and regulating the body's innate immunity, so as to assist the weakness and relieve the strong [23]. Acupuncture can play a two-way regulatory role in gastrointestinal tract, and has its special advantages in the treatment of acute and critical patients [24]. First, acupuncture therapy is simple, convenient, and low-cost, which can greatly reduce the medical burden of patients and society, with high clinical feasibility. Secondly, acupuncture therapy does not need to be absorbed through gastrointestinal tract, which reduces the burden of gastrointestinal tract. Our study applied ultrasonography to assess the effect of acupuncture on the contraction area of gastric antrum in patients, and found that before acupuncture, the contraction area of the gastric antrum was increased. After acupuncture for two days, the contraction area of the gastric antrum was decreased compared with that before acupuncture treatment. After acupuncture for five days, the contraction area of the gastric antrum was further decreased and was basically restored to a normal condition. Moreover, after treatment, the maximal pressure and maximal volume of the two groups both increased, and the study group increased more. As far as we know, HF, LF, and VLF are widely accepted as markers of the autonomic nervous functions [25]. Based on this, our study found acupuncture could adjust the downward trend of vagus nerve tension and the upward trend of sympathetic nerve tension caused by gastric distention, so as to improve vagus nerve tension and reduce sympathetic nerve tension. In addition, gastric residual, intra-abdominal pressure was decreased, and gastric compliance was improved in both groups after treatment. In addition, the recovery of gastric function in the study group was more significant than that in the control group [26]. The above data show that acupuncture can promote intestinal peristalsis, improve gastrointestinal rhythm, and restore gastric motility in patients with sepsis GD. Furthermore, the APACHE II score, WBC, CRP, and RCT of the two groups after treatment were lower than those before treatment, indicating that the treatment of the two groups had an improvement effect. However, there was no significant difference in WBC, CRP, and RCT between the two groups after treatment. Considering that the decrease of inflammation level between the two groups is more likely related to comprehensive treatment such as anti-infection, fluid resuscitation, clearance of inflammatory mediators, mechanical ventilation, and organ function support. Finally, although the abdominal circumference of the two groups did not change much before and after treatment, it cannot be completely denied that the treatment did not reduce the effect of abdominal circumference; it may also be related to the edema changes of patients before and after treatment.

RETRACTED

However, there are limitations in the study. First, the sample size was relatively small in the study. More studies should be conducted in the future. Second, the trial lacked a sham acupuncture control group because most of the Chinese patients had been treated with acupuncture and it was difficult to blind the subjects.

## 5. Conclusion

The clinical application of acupuncture in the treatment of sepsis patients with GD can significantly reduce gastric residual, abdominal pressure, improve abdominal distension, promote gastrointestinal peristalsis and gastric motility, and restore gastrointestinal autonomic nerve function. In the early stage of sepsis, abdominal distension, vomiting, intestinal dyskinesia, and more gastric residue can be used as appropriate.

## Figures and Tables

**Figure 1:** Ultrasonogram of GD at different time points. (a) Before acupuncture, result of ultrasonography indicates the increased contraction area of the gastric antrum. (b) After acupuncture for two days, result of ultrasonography indicates the decreased contraction area of the gastric antrum compared with that before acupuncture treatment. (c) After acupuncture for five days, result of ultrasonography indicates that the contraction area of the gastric antrum was decreased compared with that before acupuncture treatment and was basically restored to a normal condition.

**Figure 2:** Delayed gastric emptying (gastric residual volume) from the day before treatment to the sixth day after treatment with gastrointestinal motility drugs (control group) and acupuncture (study group). Acupuncture caused a smaller gastric residual volume. ^###^*P* < 0.001, days 0-6 vs. day -1, ^∗∗^*P* < 0.01, ^∗∗∗^*P* < 0.001, control group vs. study group.

RETRACTED

**Table 1:** Comparison of the initial and maximal pressure and volume between the two groups.

Observed indexes	Control group (*n* = 36)		Study group (*n* = 37)	
	Before treatment	After treatment	Before treatment	After treatment
Initial pressure (mmHg)	4.62 ± 1.06	6.15 ± 1.61^∗^	4.84 ± 1.24	8.44 ± 1.93^∗^^,#^
Initial volume (ml)	302.20 ± 36.41	401.34 ± 56.85^∗^	297.11 ± 33.37	492.32 ± 54.68^∗^^,#^
Maximal pressure (mmHg)	9.19 ± 1.81	12.51 ± 1.86^∗^	9.65 ± 1.79	13.69 ± 2.11^∗^^,#^
Maximal pressure (ml)	425.08 ± 76.662	693.43 ± 80.86^∗^	433.45 ± 49.76	820.71 ± 77.43^∗^^,#^

Note: ^∗^ meant *P* < 0.05 vs. before treatment; ^#^ meant *P* < 0.05 vs. after treatment in control group.

**Table 2:** Comparison of symptom scores under different gastric dilatation volumes between the two groups.

Observed indexes	Control group (*n* = 36)		Study group (*n* = 37)	
	Before treatment	After treatment	Before treatment	After treatment
Epigastric pain				
200 ml	0.94 ± 0.23	0.72 ± 0.45	0.95 ± 0.23	0.05 ± 0.23^∗^^,#^
300 ml	1.86 ± 0.76	1.06 ± 0.47^∗^	1.62 ± 0.72	0.62 ± 0.49^∗^^,#^
400 ml	2.42 ± 0.65	1.47 ± 0.65^∗^	2.27 ± 0.80	1.00 ± 0.08^∗^^,#^
Fullness				
200 ml	1.08 ± 0.28	0.97 ± 0.17	1.14 ± 0.35	0.30 ± 0.46^∗^^,#^
300 ml	1.97 ± 0.70	1.33 ± 0.79^∗^	1.65 ± 0.86	0.862 ± 0.48^∗^^,#^
400 ml	2.39 ± 0.69	1.89 ± 0.68^∗^	2.49 ± 0.61	1.32 ± 0.67^∗^^,#^
Nausea or vomiting				
200 ml	1.00 ± 0.24	0.67 ± 0.48	0.97 ± 0.29	0.11 ± 0.31^∗^^,#^
300 ml	1.78 ± 0.68	1.14 ± 0.59^∗^	1.92 ± 0.80	0.65 ± 0.54^∗^^,#^
400 ml	2.19 ± 0.82	1.44 ± 0.69^∗^	1.95 ± 0.81	0.97 ± 0.50^∗^^,#^

Note: ^∗^ meant *P* < 0.05 vs. before treatment; ^#^ meant *P* < 0.05 vs. after treatment in control group.

**Table 3:** Comparison of gastric compliance between the two groups.

	Before treatment	After treatment	*t*	*P*
Control group (*n* = 36)	45.55 ± 13.20	55.31 ± 13.99^∗^	3.043	0.0033
Study group (*n* = 37)	45.78 ± 14.96	68.45 ± 17.11^∗^^,#^	6.067	<0.0001
*t*	0.0695	3.587		
*P*	0.9448	0.0006		

Note: ^∗^ meant *P* < 0.05 vs. before treatment; ^#^ meant *P* < 0.05 vs. after treatment in control group.

**Table 4:** Effect of acupuncture on autonomic nervous function in patients with septic GD.

Observed indexes	Control group (*n* = 36)			Study group (*n* = 37)		
	Baseline	Before treatment	After treatment	Baseline	Before acupuncture	After acupuncture
HF (ms^2^)	615.1 ± 214.8	345.1 ± 132.1^∗^	299.1 ± 108.9^∗^	662.6 ± 209.9	357.7 ± 162.8^∗^	608.9 ± 308.0^#^
LF (ms^2^)	601.0 ± 221.8	798.4 ± 250.7^∗^	788.7 ± 207.9^∗^	546.8 ± 248.0	888.1 ± 320.5^∗^	600.7 ± 168.7^#^
VLF (ms^2^)	1497.1 ± 482.5	2038.4 ± 503.0^*^	1891.2 ± 369.4^*^	1401.3 ± 453.9	1893.4 ± 440.0^*^	1459.6 ± 438.3^#^

Note: ^∗^ meant *P* < 0.05 vs. baseline; ^#^ meant *P* < 0.05 vs. before acupuncture.

RETRACTED

**Table 5:** Comparison of APACHE II score, abdominal circumference, and intraperitoneal pressure between the two groups.

Observed indexes	Control group (*n* = 36)		Study group (*n* = 37)	
	Before treatment	After treatment	Before treatment	After treatment
APACHE II score	21.08 ± 2.38	16.36 ± 2.69^∗^	21.16 ± 2.21	14.62 ± 1.46^∗^^,#^
Abdominal circumference (cm)	109.62 ± 8.37	106.12 ± 7.82	109.5 ± 7.99	105.08 ± 7.55
Intraperitoneal pressure (mmHg)	14.66 ± 1.24	12.48 ± 2.11∗	14.87 ± 1.33	10.63 ± 1.62∗,#

Note: ∗ meant *P* < 0.05 vs. before treatment; # meant *P* < 0.05 vs. after treatment in control group.

**Table 6:** Comparison of infection indexes between the two groups.

Observed indexes	Control group (*n* = 36)		Study group (*n* = 37)	
	Before treatment	After treatment	Before treatment	After treatment
WBC (×10^9^/l)	14.03 ± 2.43	8.35 ± 0.76^∗^	14.80 ± 2.30	8.43 ± 0.97^∗^
CRP (mg/l)	127.92 ± 26.67	34.73 ± 10.44^∗^	127.92 ± 29.14	37.05 ± 12.50^∗^
PCT (ng/ml)	8.07 ± 1.59	2.02 ± 0.57^∗^	8.10 ± 1.52	1.94 ± 0.57^∗^

Note: ^∗^ meant *P* < 0.05 vs. before treatment.

## Data Availability

Data are available from the corresponding author under reasonable requests.
